RETRACTED

# Experimental Research on Badminton Teaching of Physical Education Major Based on Deep Learning in the Multimedia Environment

**DOI:** 10.1155/2022/9249635

**Published:** 2022-03-16

**Authors:** Shuaiyu Lian

**Affiliations:** Faculty of Education, SEGi University, Selangor 43200, Malaysia

## Abstract

There are many problems in the routine badminton teaching; there are mainly three aspects in college teaching. One is that the hardware equipment related to badminton is not enough; the second is that the badminton teaching does not meet the educational goals; the third is that the participation of college students is not high, which is no longer suitable for the current practical teaching. In order to improve the teaching method of badminton and improve the students' special performance of badminton, this paper studies the teaching of badminton based on multimedia environment. 82 students majoring in badminton were randomly divided into two classes. The experimental class (*n* = 41) used multimedia badminton teaching, and the control class (*n* = 41) used traditional badminton teaching, which lasted for one semester. Before and after the experiment, the students' physical fitness and badminton performance were tested. And the two classes of students were to send questionnaires to investigate interest in learning badminton and teaching satisfaction. The results of standing long jump, 50 m, and 800 m of the experimental class were improved by 0.2 m, 1.13s, and 16.25s, respectively. This shows that the physical quality and badminton performance of the experimental class under the multimedia environment are better than those of the control class under the general teaching. In the experimental class, 16 students are very interested in learning badminton, and 22 students are very satisfied with the multimedia teaching method; in the control class, only 9 students are very interested in learning badminton, and only 13 students are very satisfied with the traditional teaching method, which shows that the interest and satisfaction of students in the experimental class under the multimedia environment are higher than those in the control class under the traditional teaching.

## 1. Introduction

### 1.1. Background Significance

In the era of highly informatized and fragmented knowledge economy, the basic feature of the era of fragmentation is the fragmentation of information. The massive simplification and segmentation of the process have led to incomplete information and internal logic. The fast-paced life makes people's time fragmented, which affects the way people learn. People's learning methods, learning paths, and learning tasks have undergone major changes, and society has also put forward new requirements for human training. The traditional classroom teaching of “full classroom” or “one-word classroom” hinders the development of students' deep learning. The traditional classroom teaching model is unidirectional indoctrination, students are in a passive state of acceptance, and the initiative of learning is ignored or even suppressed. Under the background of the new era, as the goal pursued by education and teaching, deep learning requires teaching to shift from inherent knowledge to the cultivation of learners' deep learning ability. Under the trend of in-depth integration of information technology and classroom teaching, this is because the focus of deep learning is to cultivate children's metacognitive ability, critical thinking, creative thinking, problem awareness, and problem solving skills and other high-level development of abilities, so that they can critically learn new knowledge. How to effectively achieve deep learning and develop deep learning with the support of information technology has become an important proposition for the development of education. It promotes the blended teaching of deep learning; that is, according to the goal of deep learning, through the method of blended teaching, it refers to a teaching model that combines the advantages of online teaching and traditional teaching, combining “online” and “offline.” Through this mode, learners' learning can be guided from shallow to deep to deep learning to promote students to achieve deep learning and cultivate students' deep learning ability. At the same time, deep learning theory and blended learning theory are integrated to jointly guide blended teaching design. The forms of blended teaching are diversified, and everything is taught for the realization of deep learning.

RETRACTED

With the wide spread of multimedia network, it is imperative to reform the physical education curriculum by combining multimedia technology with physical education. Badminton teaching should not only learn the basic action essentials, but also cultivate students' aesthetic feeling and integrate sports and art. In the traditional badminton teaching, because there is no complete comprehensive training system, the speed of students mastering the technical essentials is slow, unable to complete the teaching task. Through multimedia technology to integrate teaching resources, let students master more abstract action essentials, establish their own knowledge system, and improve teaching efficiency [1]. This is the focus of contemporary badminton teaching. There are few researches on the use of multimedia in badminton teaching. This study provides a theoretical basis for related teaching and curriculum reform.

### 1.2. Related Work

Armenteros M aims to enhance the understanding of the different behavioral intentions of different FIFA referees and assistant referees regarding multimedia teaching materials as learning tools. In order to achieve this goal, they investigated 214 excellent referees and assistant referees [2]. Feng S designs a video conversion system based on SOPC and finally constructs a multimedia teaching system based on multifunctional video conversion from two aspects of module design and function design and tests the learning effect of college students' basketball class by using a randomized controlled experiment [3].

Badminton needs a high level of flexibility, conditioning, and complete body complement, which is rarely comparable to other sports. Leandro C aims to analyze the difficulty judgment quality of badminton at different performance levels, and the sample includes 1152 difficulty scores. In the validity evaluation, he calculated the average deviation of judges' difficulty score, Kendall consistency coefficient W, and the square value of analysis of variance ETA [4]. The research of the above-mentioned scholars has a certain representative significance in a comprehensive view, but most of the research contents are not easy to obtain experimental samples, or the selection of samples is biased and cannot represent the whole, and the process is more complicated. In summary, their research results provide the reference of experimental methods and the support of theoretical basis for the research of this paper.

### 1.3. Innovative Points in This Paper

The innovations of this paper are as follows: (1) apply multimedia technology to badminton teaching, and put it into practical teaching. (2) In this paper, a comparative experiment between multimedia badminton teaching and traditional badminton teaching is carried out, and the pretest and posttest are carried out to analyze the changes of students' physical fitness and badminton performance under different teaching methods. (3) Through the investigation of students' learning interest and teaching satisfaction, it is proved that multimedia teaching method is helpful to improve students' learning interest and satisfaction.

## 2. Multimedia Environment and Rhythmic Gymnastics Teaching

### 2.1. Multimedia Teaching Technology

#### 2.1.1. Stage of Multimedia Teaching Technology

Multimedia teaching means that, in the teaching process, according to the characteristics of teaching goals and teaching objects, through teaching design, rational selection and use of modern teaching media, and organic combination with traditional teaching methods, jointly participate in the whole teaching process. Tracing back to the source, no matter how advanced multimedia-assisted teaching is, it is closely related to program teaching methods.

RETRACTED

Program teaching and teaching machine are the basis of multimedia teaching. Program teaching is a teaching method that uses program teaching materials automatically. Divide the teaching materials into a certain order. The learner will answer, and the answer is correct, and then he will enter the next learning project. If the correct answer is not possible within the limit, the correct answer or prompt will be displayed to promote their learning. The more excellent multimedia-assisted learning software mostly adopts the idea of program teaching; the teaching process is carried out by teaching machines. It is equipped with program teaching materials, which can display problems to learners according to the program, analyze learners' responses, and point out right and wrong. One of the important trends of school teaching information development is network. The development of computer teaching can be divided into several stages from theory, technology, and development methods [5, 6]. The first stage is the development of computer hardware, which mainly combines some output and input devices with the computer to make it a specific teaching aid machine. Then we step into the stage of computer language development, mainly using the developed programming language to achieve complex teaching simulation.

Based on the three basic characteristics of multimedia technology: first, vivid and realistic sound effects; second, colorful dynamic video; third, flexible and convenient interactive means, these three characteristics can effectively attract learners to study, so multimedia-assisted teaching is valued. Multimedia have the advantages of large information content and strong expression, and multimedia-assisted teaching has been paid attention to. Finally, at this stage, it is based on the development stage of network application, with the characteristics of networking and globalization of teaching resources [2]. The field of educational technology is also influenced and infiltrated by constructivist learning theory, especially the design of learning environment, which fully embodies the basic concepts and ideas of constructivist learning theory.

The development of multimedia teaching has experienced three important turns, the first is the computer from programming to auxiliary teaching [7], as shown in Figure 1. With the computer-aided instruction gradually exposing fixed procedures and closed problems, it began to become unsuitable for the reality of classroom teaching. In order to better adapt to the development of network education, multimedia teaching has changed from standalone courseware to web-based courseware or integrable ware.

RETRACTED

#### 2.1.2. Advantages of Multimedia Teaching

The emergence of network technology and multimedia platform can enrich the means and methods of teaching. The transmission of teaching information is no longer limited to classroom teaching and teachers' teaching, and the media platform has also become the medium of teaching communication [8]. Students can use the terminal platform to receive teaching information and practice after class.

Multimedia teaching can improve the effect of students' extracurricular exercises. In their spare time, students can review the key points in class through video and other forms of learning resources, carry out more targeted exercises, and improve the effect of after-class exercises. According to the classroom performance, students can be urged to review and consolidate the learning content after class.

The application forms of multimedia in teaching include classroom teaching mode, individualized autonomous learning mode, and distance education mode [9]. Classroom teaching mode belongs to the demonstration teaching; teachers control the media equipment to achieve the teaching purpose. Individualized autonomous learning mode mainly provides students with a platform for autonomous learning. Teachers and students can achieve the teaching purpose through human-computer interaction and online dialogue. Distance education mode uses network to realize distance education. Teachers and students can consult materials, practice, and study.

Generally speaking, for its specific characteristics, the first is comprehensive performance, including the compatibility of information dissemination technology equipment. The second is real-time controllability, real-time service for needs. The third is interactive applicability, a way of active learning based on needs. The fourth is dynamic presentation, which increases the interest of learning and reduces the difficulty of learning. The key to using computer multimedia to assist teaching is to fully apply these characteristics to serve our teaching.

### 2.2. Badminton Teaching

Deep learning and deep teaching have not substantially promoted the change of classroom teaching, and deep learning and deep teaching have not been substantively implemented in the actual progress of classroom teaching. The deep learning and deep teaching in the current teaching practice have not really entered the hearts of students and have not really attracted teachers and students' attention, and students have not really understood the concept of deep learning on the ideological level. The general architecture of deep learning is shown in Figure 2.

RETRACTED

#### 2.2.1. Problems in Traditional Badminton Teaching

In the traditional badminton special syllabus and teaching plan, when cultivating students' badminton ability and comprehensive ability, there are no specific and detailed plan steps for ability training. In this way, it is impossible to reflect the specific effect of the curriculum on the cultivation and development of students' abilities [10]. In terms of content, there is also a lack of hierarchy and comprehensiveness, and it is impossible to systematically build students' badminton skills.

In the actual teaching of badminton, the distribution of the teaching content of student ability building is relatively random, there is no complete scientific hierarchical classification ability system, and the teaching process does not follow the principle of gradual progress. When evaluating the level of student's ability development, it is only based on classroom performance and test results, the focus of teaching management also stays in the classroom, and very few extracurricular activities and practical activities are organized.

The content of the traditional badminton teaching evaluation mechanism is not detailed and specific enough. It pays attention to academic performance, which can easily lead to one-sided evaluation and error [11]. A complete teaching evaluation system should evaluate students' teaching training, cognitive level, and learning attitude in many aspects.

#### 2.2.2. Factors Affecting the Teaching of Badminton

School education factor is an important factor affecting badminton teaching. The teaching environment of badminton is poor, the popularity rate in the country is low, and the participation of students is not high. The decrease in the number of people engaged in artistic gymnastics teaching and the inability of the material basis of venues to keep up with it will also directly affect the teaching of badminton, and the teaching plan cannot be implemented [12].

Social factors will also have a certain impact on badminton teaching. The society's change in the value of measuring talents has gradually increased people's demand for sports. There is a contradiction between the remuneration of badminton teachers and the value of their talents. Some teachers are not mindful of their own work and did not give full play to their actual teaching level in the teaching process. This has caused a great negative impact on the development of badminton teaching [13].

Students' sports values will also affect the teaching of badminton. People have misunderstandings about badminton, thinking that it is difficult and demanding, and it is a difficult art sport [14]. Over time, the distance between everyone and badminton is getting farther and farther, and there is less and less need for badminton learning. Such one-sided sports values will directly affect the effectiveness of badminton teaching.

RETRACTED

#### 2.2.3. Principles of Badminton Teaching

First of all, we must follow the principles of planning and gradualism. The teaching of badminton cannot be done quickly. It needs to be gradual and develop certain training goals and plans [15, 16]. Link to the actual teaching process, formulate specific teaching measures that can be implemented, and cultivate students' badminton ability in a purposeful and planned manner.

Second, we must follow the principle of comprehensiveness and combine theoretical knowledge with practice. When cultivating students' badminton ability, according to the actual situation of each stage, effectively combine badminton courses and other courses [17]. It can also allow students to make suggestions and adjustments to the teaching content to improve their abilities in practice.

Finally, we must follow the principle of practicality. Mastering physical education knowledge and skills is the basis and condition for cultivating teaching ability, and teaching practice is the main way to cultivate teaching ability. Learn and master skills in practice to improve their abilities.

## 3. Rhythmic Gymnastics Teaching Experiment under the Multimedia Environment

### 3.1. Experimental Objects and Methods of Badminton Teaching

The research object of this paper is the badminton teaching under the multimedia environment, and the experimental object is the sophomores of badminton major in a university in Jiangxi Province. 82 students participated in the experiment and were randomly divided into two classes. The experimental class (*n* = 41) used multimedia badminton teaching, and the control class (*n* = 41) used traditional badminton teaching, which lasted for one semester.

Before and after the experiment, the students' physical fitness and badminton performance were tested. Compare the two classes of students' physical fitness and badminton special good performance changes, and to the two classes of students send questionnaires to investigate the interest in learning badminton and teaching satisfaction.

### 3.2. Relevant Data Capture Algorithm

BP neural network is a multilayer feedforward network trained by error backpropagation algorithm, and it is one of the most widely used neural network models. The BP network can learn and store a large number of input-output pattern mapping relationships without the need to publicly describe the mathematical equations of this mapping relationship in advance. Its learning rule is to use the steepest descent method to continuously adjust the weight and threshold of the network through backpropagation to minimize the sum of squared errors of the network.

RETRACTED

BP neural network algorithm is used to calculate the relevant data of badminton major students in our school. The calculation of the output value of each unit in the hidden layer is shown in the following:

(1) $$\begin{array}{c} y_{j}=f\left(\sum_{i=1}^{n}u_{ij}x_{i}-s_{j}\right). \end{array}$$

The threshold value in the neuron model is written into the join weight, so that *u*_0*j*_=−*s*_*j*_, *x*_0_=−1. Formula 1 can be transformed into

(2) $$\begin{array}{c} y_{j}=f\left(\sum_{i=0}^{n}u_{ij}x_{i}\right). \end{array}$$

The calculation formula is shown in the following:

(3) $$\begin{array}{c} O_{k}=f\left(\sum_{j=1}^{m}z_{ij}y_{j}-s_{k}\right). \end{array}$$

Similarly, if *z*_0*k*_=−*s*_*k*_, *y*_0_=−1, (3) is changed into the following:

(4) $$\begin{array}{c} O_{k}=f\left(\sum_{j=0}^{m}z_{jk}y_{j}\right). \end{array}$$

The fourth step is to calculate the difference between the actual output value and the expected output value and judge whether the difference is less than the previously set error range. If it is less than it, select the next sample to continue training; if it is greater than it, carry out error backpropagation and adjust the weight to reduce the difference. The weight correction of output layer is shown in the following:

(5) $$\begin{array}{c} \Delta z_{ij}=-\mu \frac{\partial E}{\partial z_{ij}}\\ =-\mu \frac{\partial E}{\partial {\text{net}}_{k}}\cdot \frac{\partial {\text{net}}_{k}}{\partial z_{ij}}. \end{array}$$

The fifth step is to skip to the next sample pair in order and continue training until all samples have completed the training. The sixth step is to import the new samples into the neural network for testing after the training of all samples.

## 4. Discussion on the Experimental Results of Badminton Teaching

### 4.1. Comparison of Physical Fitness before and after the Experiment

Physical fitness test items include standing long jump, 50 m, and 800 m.

As shown in Table 1, after the experiment, the standing long jump score of the experimental class was 2.02 ± 0.13 M and that of the control class was 1.93 ± 0.18; the 50 m score of the experimental class was 8.15 ± 0.2 s and that of the control class was 8.71 ± 0.33 s; the 800 m score of the experimental class was 141.13 ± 8.26 s and that of the control class was 148.69 ± 9.13 s. This shows that the physical quality of the experimental class under the multimedia environment is better than that of the control class under the ordinary teaching.

RETRACTED

As shown in Figure 3, the physical fitness of the two classes before and after the experiment has been improved. The results of standing long jump in the experimental class increased by 0.2 m, 1.13 s in 50 m, and 16.25 s in 800 m. The results of standing long jump in the control class increased by 0.12 M, 50 m by 0.36 s, and 800 m by 10.43 s.

### 4.2. Comparison of Badminton Performance before and after the Experiment

Before and after the experiment, the badminton scores of the two classes were tested. The badminton score = 70% gymnastics +30% basic knowledge.

As shown in Table 2, there is no significant difference in the comprehensive score of badminton between the two classes before the experiment. After the experiment, the comprehensive score of the experimental class was 7.07 points higher than that of the control class. This shows that the performance of badminton in the experimental class is better than that in the control class.

As shown in Figure 4, the badminton scores and basic knowledge scores of the two classes before and after the experiment have been improved. The badminton performance of the experimental class was improved by 12.8 points, and the basic knowledge performance was improved by 24.7 points. The results of badminton in the control class increased by 4.2 points, and the results of basic knowledge increased by 16 points.

Badminton results are divided into singles, doubles, receiving, and serving, each accounting for 1/4.

As shown in Figure 5, the results of free hand combination, ball exercise, rope exercise, and circle exercise in the experimental class were 6.5, 2.8, 6.5, and 7.8 points higher than those in the control class. The total score of badminton in the experimental class was 84.2 points, while that in the control class was 78.3 points, with a difference of 5.9 points.

### 4.3. Questionnaire Results

At the end of the experiment, two classes of students were given questionnaires to investigate their interest in learning badminton and teaching satisfaction. The interest in badminton of the two classes can be divided into 1–5, which are very interested, relatively interested, average, not very interested, and not interested at all.

As shown in Figure 6, students in the experimental class are very interested in learning badminton, 12 students are more interested, and only 2 students are not interested at all. In the control class, only 9 students are very interested in learning badminton, 13 students are more interested, and 4 students are not interested at all.

The overall satisfaction of the class teaching methods can be divided into A to D, which are very satisfied, satisfied, general, and dissatisfied.

RETRACTED

As shown in Figure 7, students in the experimental class are very satisfied with the multimedia teaching method. It accounts for 53.7% of the total number of experimental classes, accounting for more than half, and only one student is not satisfied. In the control class, only 13 students were satisfied with the traditional teaching method, accounting for 31.7% of the control class, and 3 students were not satisfied. On the whole, the experimental class's agreement with multimedia teaching methods reached 82.9%, while the control class's agreement with traditional teaching methods was 68.3%.

## 5. Conclusions

The evaluation of students' deep learning performance is an important indicator for evaluating the effect of blended teaching in promoting deep learning. Judging from the degree of recognition of the experimental results, for the same number of people, the degree of recognition of the experimental class is 14.6% higher than that of the control class. It can be clearly seen that deep learning is currently an important learning method for improving students' learning but students' learning cannot be separated from the guidance of teachers. Teachers can better promote students' deep learning only by in-depth teaching. The emergence of network technology and multimedia platform can enrich the means and methods of teaching. The transmission of teaching information is no longer limited to classroom teaching and teachers' teaching, and the media platform has become the medium of teaching communication. Students can use the terminal platform to receive teaching information and practice after class. Through multimedia technology to integrate teaching resources, students can master more abstract action essentials, establish their own knowledge system, and improve teaching efficiency. The experimental results show that the application of multimedia technology in badminton teaching can effectively improve students' physical fitness and badminton performance and enhance students' interest and satisfaction in badminton. The results provide theoretical basis for related teaching and curriculum reform [18].

## Figures and Tables

**Figure 1:** Multimedia teaching.

**Figure 2:** Deep learning and teaching of badminton.

**Figure 3:** Comparison of physical fitness before and after the experiment.

**Figure 4:** Comparison of badminton results.

**Figure 5:** Distribution of badminton results.

**Figure 6:** Interest in learning badminton.

**Figure 7:** Satisfaction survey results.

**Table 1:** Comparison of physical fitness of two classes.

Class	Standing long jump	50 m	800 m
Experimental class B	1.82 ± 0.23	9.28 ± 0.37	157.38 ± 9.31
Control class B	1.81 ± 0.19	9.17 ± 0.41	159.12 ± 9.87
Experimental class A	2.02 ± 0.13	8.15 ± 0.2	141.13 ± 8.26
Control class A	1.93 ± 0.18	8.71 ± 0.33	148.69 ± 9.13

RETRACTED

**Table 2:** The difference of teaching effect between the two classes.

Class	Gymnastics	Basic knowledge	Comprehensive
Experimental class B	71.4 ± 16.3	54.8 ± 13.7	66.42
Control class B	74.1 ± 13.6	53.7 ± 14.1	67.98
Experimental class A	84.2 ± 8.3	79.5 ± 9.2	82.79
Control class A	78.3 ± 9.8	69.7 ± 10.1	75.72

## Data Availability

No data were used to support this study.
